# KIF11 Is a Promising Therapeutic Target for Thyroid Cancer Treatment

**DOI:** 10.1155/2022/6426800

**Published:** 2022-08-16

**Authors:** Yue Han, Jing Chen, Dianjun Wei, Baoxi Wang

**Affiliations:** ^1^Department of Clinical Laboratory, The Secondary Hospital of Tianjin Medical University, Tianjin, China; ^2^Department of Pancreatic Cancer, Tianjin Tumor Hospital, Tianjin, China; ^3^Department of Clinical Laboratory, Hebei Yanda Hospital, Yanda International Health City, Sibilan Road, Yanjiao Economic and Technological Development Zone, Langfang, 065201 Hebei Province, China

## Abstract

**Objective:**

To assess KIF11 expression in human thyroid tumor tissues and further evaluate its involvement in thyroid cancer.

**Methods:**

The expression of KIF11 in 71 cases of thyroid carcinoma as well as corresponding tissues was detected by the immunohistochemical (IHC) method. Patients were divided into the high KIF11 expression as well as low expression groups based on the staining levels. In addition, to study the relationship between the expression of KIF11 as well as clinicopathological features, the effects of KIF11 were detected on the proliferation, apoptosis, and cell cycle of two types of thyroid cancer cells, TPC-1 and KTC-1, through colony formation assays, MTT assays, and FCM assays, respectively. We further assessed the potential effects of KIF11 on tumor growth using an animal model.

**Results:**

The significantly high expression of KIF11 in thyroid tumor tissues was revealed, and the correlations between KIF11 expression levels as well as clinical pathological features (T stage and intraglandular dissemination) of patients were revealed. We further noticed that KIF11 knockdown remarkably suppressed thyroid cancer cell proliferation as well as induced cell apoptosis of thyroid cancer cells. Additionally, KIF11 contributed to tumor growth of thyroid cancer cells in mice.

**Conclusions:**

We noticed the involvement of KIF11 in the progression of thyroid cancer.

## 1. Introduction

Thyroid cancer accounts for 1% of all malignant tumors in the body [1], with low malignancy as well as slow progression [2, 3]. However, its growth rate is among the highest among all solid tumors [4–6]. For metastatic thyroid cancer, the existing treatment methods cannot meet the clinical needs, while targeted therapy shows strong advantages [7]. Several targeted therapeutic drugs, such as vandetanib and sorafenib, have been used to treat this type of cancer [8], whereas more effective therapeutic targets are urgently needed.

Kinesin family member 11 (KIF11) is a molecular motor protein involved in many cellular processes [9, 10]. KIF11 could affect the separation of centrosomes as well as the formation of the spindle [11, 12]. In addition, a previous study indicated that the depletion of KIF11 led to cell division defects and cell cycle arrest, so as to induce the apoptosis of cells [13]. As was known, KIF11 affected cell migration through the regulation of axonal branching and growth cone motility in a non-mitosis-dependent manner [14].

KIF11 affected the prognosis of multiple types of cancers [15–18]. The inhibitor of KIF11, K858, could induce apoptosis and also survivin-related chemoresistance in breast cancer cells [19]. In addition, several compounds that inhibit KIF11 have entered Phase I or II clinical trials as monotherapies [19]. Although KIF11 plays a critical role in a variety of tumors, its potential effects on thyroid cancer remain unclear.

This study was aimed at investigating the expression of KIF11 in thyroid cancer tissues and clarifying its effects on the progression of thyroid cancer. We found that KIF11 was highly expressed in human thyroid cancer tissues. KIF11 knockdown remarkably suppressed thyroid cancer cell proliferation as well as induced cell apoptosis of thyroid cancer cells, suggesting that KIF11 may be a potential therapeutic target for thyroid cancer.

## 2. Materials and Methods

### 2.1. Antibodies, Primers, and Plasmids

Antibodies used are anti-KIF11 antibody (for immunohistochemical, 1 : 100 dilution, for immunoblot, 1 : 1000 dilution, ab5694, Abcam, Cambridge, UK) and anti-*β*-actin (1 : 2000 dilution, ab8226, Abcam, Cambridge, UK).

Ready-to-package AAV shRNA clone for KIF11 was bought from Addgene; the targeted sequences were as follows: 5′-AATAGTAGAATGTGATCCTGTAC-3′.

### 2.2. Human Tissue Samples and IHC Assays

A total of 71 human thyroid cancer tissues and adjacent nontumor tissues were collected from the patients receiving surgical resection in our hospital from September 2012 to May 2022 (Table 1). Tumor tissues were isolated from mice in the tumor growth assays.

Sample sections were fixed with 4% PFA for 25 min and subsequently blocked with 2% BSA for 20 min. Sections were incubated with KIF11 antibodies for 2 h. Subsequently, the slices were incubated with biotin-labeled secondary antibody for 1.5 h, and diaminobenzidine was used as a chromogen substrate.

### 2.3. Cell Culture and Transfection

TPC-1 and KTC-1 human thyroid cancer cells were bought from ATCC. TPC-1 cells were maintained in high-glucose DMEM culture medium (Gibco, USA), and KTC-1 cells were maintained in F-12K culture medium (Gibco, USA), respectively, with 10% of fetal bovine serum at 37°C in a 5% CO_2_ incubator.

### 2.4. Quantitative PCR Assay

This experiment was performed according to the previous study [20]. The TRIzol reagent (15596026, Invitrogen, Carlsbad, CA, USA) was used to extract total RNA. Then, the total RNA was reverse-transcribed by M-MLV (M1701, Promega, Wisconsin, USA).

Total RNA was reverse-transcribed to produce cDNA by the cDNA synthesis system. KIF11 expression was normalized to that of GAPDH.

### 2.5. Immunoblot Assays

This experiment was performed according to the previous study [20]. Cells or tissues were lysed in RIPA Buffer (9800, Cell Signaling, MA). Then, the samples were analyzed with 8% SDS-PAGE. Subsequently, the polyvinylidene fluoride (PVDF) membranes were blocked with 5% milk and then incubated with the primary antibodies as well as HRP-conjugate secondary antibodies for 2 h, respectively. Signals were visualized with an ECL kit.

### 2.6. Colony Formation Assays

Approximately 500 TPC-1 and KTC-1 cells were seeded per well (6-well plate). The medium was refreshed every 3 days. After 14 days, cells were fixed with methanol as well as stained with 0.1% crystal violet for 30 min and washed.

### 2.7. MTT Assays

Thyroid cancer cells were plated into 96-well plates with a density of about 1000 cells each well. Cells were then incubated with MTT for 4 h and removed. Then, 150 *μ*L dimethyl sulfoxide (DMSO) was added, and the OD570 value was measured.

### 2.8. Cell Cycle Assays

Thyroid cancer cells were fixed with 70% ethyl alcohol for 24 h at -20°C and incubated with 50 *μ*g/mL propidium iodide (PI) at 37°C for 30 min; then, the samples were analyzed using FACS (Beckman Coulter, CA).

### 2.9. Cell Apoptosis Assays

Cells were resuspended in 100 *μ*L binding buffer with 5 *μ*L of annexin V-FITC and incubated for 10 min. Subsequently, 5 *μ*L of PI solution was added, and cells were incubated for another 5 min.

### 2.10. Tumor Growth Assays

All animal assay processes were approved by the Animal Ethical and Welfare Committee (AEWC) in Tianjin key laboratory of radiation medicine and molecular nuclear medicine (SYXK-2019-0002). TPC-1 cells were stably transfected with control or KIF11 shRNA. Then, approximately 2∗10^6^ cells were subcutaneously implanted into athymic nude mice. After 2 weeks, tumors began to be formed and then were isolated, and the volume was measured every 3 days.

### 2.11. Statistics

GraphPad Prism 5.0 software (GraphPad, USA) was used. All data were represented as the mean ± standard deviation (SD). The correlation between clinical data and KIF11 expression was calculated using *χ*^2^ analysis. ∗ indicates *p* < 0.05 and is considered significant.

## 3. Results

### 3.1. KIF11 Was Highly Expressed in Human Thyroid Tumor Tissues

To explore the expression and the performance of KIF11 in thyroid cancer patients, we first detect the expression of KIF11 in different types of cancers. We noticed the high expression of KIF11 in several types of cancers (Figure 1). The mRNA levels of KIF11 were also obviously high (Figure 2(a)). We further noticed that the expression of KIF11 was correlated with the disease-free survival rate of patients (Figure 2(b)).

The expression of KIF11 was detected using tumor tissues and corresponding tissues of thyroid cancer patients in our hospital. Compared with the adjacent tissues, the tumor tissues showed an obviously high KIF11 expression (Figures 3(a) and 3(b)).

### 3.2. The Clinical Significance Analysis between KIF11 Expression and the Clinical-Pathological Features of Patients with Thyroid Cancer

To conduct the analysis, a total number of 71 tumor tissue samples from patients who underwent thyroid cancer were manually classified into the KIF11 low and high expression groups based on the expression levels (Figure 3(a) and Table 1). We noticed that 14 patients exhibited low expression of KIF11, whereas 57 showed high KIF11 expression (Table 1).

We then analyzed the clinical-pathological significance between KIF2A expression and clinical features of patients. According to the results, no obvious clinical correlation was found in features including patient age (*p* = 0.153), gender (*p* = 0.192), and lymph node metastasis (*p* = 0.860) between the KIF11 low and high expression groups (Table 1). Notably, our results showed that KIF11 expression was significantly related to T stage (*p* = 0.009^∗^) and intraglandular dissemination (*p* = 0.010^∗^) (Table 1). We therefore indicated that KIF11 expression levels were associated with clinical features including T stage and intraglandular dissemination of thyroid cancer patients.

### 3.3. KIF11 Fascinates Proliferation and Suppresses Apoptosis of Thyroid Cancer Cells In Vitro

To explore the effects of KIF11 on the progression of thyroid cancer in vitro, shRNA plasmids specifically targeting KIF11 were used to deplete KIF11 in two types of thyroid cancer cell lines, TPC-1 and KTC-1 cell lines. Quantitative PCR (Figure 4(a)) and immunoblot (Figure 4(b)) assays were, respectively, performed. The transfection of KIF11 shRNA plasmids effectively decreases its expression in both TPC-1 and KTC-1 cells, respectively.

Subsequently, to explore the possible involvement of KIF11 in the proliferation of thyroid cancer cells, colony formation assays and MTT assays were performed. We found that ablation of KIF11 dramatically decreased the colony numbers of TPC-1 and KTC-1 cells, respectively (Figure 5(a)). Similarly, through MTT assays, we noticed that the OD value (570 nm wavelength) of KIF11-knockdown groups was obviously decreased after 48 hours in both TPC-1 and KTC-1 cells (Figure 5(b)).

We then performed FCM assays to detect the effects of KIF11 on the apoptosis of TPC-1 and KTC-1 cells. The ablation of KIF11 obviously induced apoptosis in TPC-1 and KTC-1 cells (Figure 5(c)). We also assessed whether KIF11 affected the cell cycle of thyroid cancer cells and revealed that KIF11 depletion obviously induced the arrest of the cell cycle in TPC-1 and KTC-1 cells (Figure 5(d)).

### 3.4. KIF11 Contributes to Tumor Growth of Thyroid Cancer Cells in Mice

Tumor growth assays were then performed. TPC-1 cells were infected with control or KIF11 shRNA lentivirus and injected into nude mice. After 2 weeks, tumors began to be formed and were isolated every 3 days and photographed, and the volume of tumors was measured. After 29 days, all tumors were isolated. Representative tumors and the growth curve are all exhibited in Figure 6(a). The volume of tumors in the KIF11 knockdown groups was significantly smaller than control (Figure 6(a)). The silencing of KIF11 in tumor tissues from the depletion groups was confirmed (Figure 6(b)).

## 4. Discussion

Advanced thyroid cancer is still challenging due to the high metastasis and the lack of effective therapy options [21, 22]. The possible role of KIF11 in the progression of cancers has been widely revealed [23]. Firstly, we found the high expression of KIF11 in thyroid cancer tissues through IHC assays. We also found the correlation between KIF11 and the clinical features of patients. Furthermore, KIF11 depletion led to proliferation inhibition, induced cell apoptosis, and the arrest of cell cycle. Our in vivo results showed that KIF11 ablation suppressed tumor growth in mice.

KIF11 was involved in the progression of multiple types of cancers [17, 23, 24]. This is similar to our results for thyroid cancer [18]. In addition, KIF11 also affected the migration of ovarian cancer cells, which was promoted by death receptor 6 (DR6) [17]. We next should detect whether KIF11 affects the migration of thyroid cancer cells.

Indeed, this therefore resulted in the arrest of cell cycle and the induction of apoptosis, which was also found in this study. Previous studies also revealed the mitosis-independent functions of KIF11, such as neuronal growth cone extension and migration, suggesting that KIF11 might affect the activity of thyroid cancer cells in multiple modes of regulation [25, 26]. However, the precise molecular mechanism underlying KIF11 promoting progression needs further study.

In addition to KIF11, other members of the KIF family could affect the progression and development of cancer; most of them could be potential cancer molecular targets [20]. A previous study indicated that KIF14 could contribute to the growth of hepatocellular carcinoma (HCC) [27]. KIF4A, KIF14, and KIF20A were shown to be highly expressed in many types of cancers [24, 28–30]. Our study investigated another member of the KIF family, KIF11, affecting the proliferation and apoptosis of thyroid cancer cells.

KIF11, a member of the cell division driver family, is involved in the formation of bipolar mitotic spindles during cell division. Studies have found that these motor proteins are widely expressed and play an important role in cell division and intracellular transport. These microtubule-associated driver proteins, due to their important biological functions in cell division, are closely related to tumor formation and are prognostic factors for a variety of malignant tumors. Therefore, KIF11 has also become a new target for tumor targeted therapy, and our in vitro and in vivo studies further confirm this conclusion.

In summary, we revealed the high expression of KIF11 in human thyroid tumor tissues. We revealed KIF11 in the progression of thyroid cancer and provide a promising therapeutic target for the treatment of thyroid cancer.

## Figures and Tables

**Figure 1:** KIF11 expression in different types of cancer tissues according to TCGA database.

**Figure 2:** KIF11 expression in tumor tissues and normal tissues according to the GEPIA database.

**Figure 3:** KIF11 was highly expressed in human thyroid tumor tissues. (a) The representative photographs of IHC assays showed the expression of KIF11 in thyroid cancer tissues (100x and 200x magnification, respectively). (b) IHC assays were performed to exhibit KIF11 expression levels in adjacent tissues, and the representative photographs are shown (100x and 200x magnification, respectively). Scale bar, 50 *μ*m.

**Figure 4:** The expression levels of KIF11 were effectively decreased in both TPC-1 and KTC-1 cells caused by the transfection of KIF11 shRNA plasmids. (a) The results of quantitative PCR assays showed the obviously decreased expression levels of KIF11 caused by the transfection of its shRNA plasmids in TPC-1 and KTC-1 cells, respectively. (b) Immunoblot assays showed KIF11 expression levels upon the transfection of control or KIF11 shRNA plasmids in both TPC-1 and KTC-1 cells. Results are presented as the mean ± SD, ^∗^*p* < 0.05.

**Figure 5:** KIF11 fascinates thyroid cancer cell proliferation and suppresses cell apoptosis in vitro. (a) Colony formation assays were conducted using TPC-1 and KTC-1 cell transfection, and the number of colonies was counted. Scale bar, 5 mm. (b) MTT assays showed the OD value at 570 nm wavelength of KIF11-depleted cells. (c) FCM assays confirmed the effects of KIF11 depletion on the apoptosis in TPC-1 and KTC-1 cells. (d) FCM assays showed that KIF11 ablation led to the arrest of cell cycle in TPC-1 and KTC-1 cells. Results are presented as the mean ± SD, ^∗^*p* < 0.05.

**Figure 6:** KIF11 promotes tumor growth of thyroid cancer in mice. (a) Tumor growth curves were shown. Scale bar, 5 mm. (b) Immunoblot assays exhibited the expression levels of KIF11 in tumors isolated from mice. Results are presented as the mean ± SD, ^∗^*p* < 0.05.

**Table 1:** Relationships of KIF11 and clinicopathological characteristics in 71 patients.

Feature	All *n* = 71	KIF11 expression		*χ* ^2^	*p*
		Low	High		
		*n* = 14	*n* = 57		
Age (year)				2.045	0.153
<45	24	7	17		
≥45	47	7	40		
Gender				1.701	0.192
Male	14	5	9		
Female	57	9	48		
T stage				6.751	0.009^∗^
T_1_-T_2_	29	10	19		
T_3_-T_4_	42	4	38		
Lymph node metastasis				0.031	0.860
Yes	34	7	27		
No	37	7	30		
Intraglandular dissemination				6.675	0.010^∗^
Yes	32	2	30		
No	39	12	27		

## Data Availability

The datasets generated during and/or analyzed during the current study are available from the corresponding authors on reasonable request.
